# Determination of volatile organic compounds exhaled by cell lines derived from hematological malignancies

**DOI:** 10.1042/BSR20170106

**Published:** 2017-06-21

**Authors:** Hongxia Tang, Yan Lu, Lulu Zhang, Zhonghui Wu, Xiaofang Hou, Hailong Xia

**Affiliations:** 1 Department of Hematology, The First Affiliated Hospital of Anhui Medical University, No. 218 Jixi Road, Hefei 230022, China; 2 Center of Medical Physics and Technology, Hefei Institutes of Physical Science, Chinese Academy of Sciences, No. 350 Shushanhu Road, Hefei 230031, China; 3 Department of Hematology, The second Affiliated Hospital of Anhui Medical University, No. 678 Furong Road, Hefei 230022, China; 4 Department of Hematology, The Chaohu Hospital of Anhui Medical University, No. 64 Northern Chaohu Road, 238000, China

**Keywords:** Acute mononuclear leukemia cell line, Exhaled gas analysis, JEOK, Non-Hodgkin's lymphoma cell line, SHI-1, Tumor

## Abstract

Background**:** The gas human exhaled contains many volatile organic compounds (VOCs), which is related to the health status of body. Analysis of VOCs has been proposed as a noninvasive diagnostic tool for certain cancers. Detailed research on the VOCs in gas exhaled by cell can characterize cell type specific metabolites and may be helpful to detect the cancer markers in clinical practice.

Methods**:** Solid-phase microextraction (SPME) gas chromatography–mass spectrometry was used to detect VOCs in the headspace of tissue culture flask in non-Hodgkin’s lymphoma (NHL) cell line JEKO and acute mononuclear leukemia cell line SHI-1, to elaborate the characteristic gaseous biomarkers of hematological malignancies. While macrophage cells and lymphocytic cells were acted as control. The blank group was only the RPMI 1640 medium containing 10% fetal calf serum that without cells.

Results**:** Comparing with control group, the concentration of dimethyl sulfide, 2,4-dimethylheptane, methylbenzene, *o*-xylene, dodecane, and 1,3-di-tert-butylbenzene in JEKO cells was relatively higher, while the concentration of ethanol, hexanal, and benzaldehyde was lower. In SHI-1 cells, the levels of 2,4-dimethylheptane, benzene, 4-methyldecane, chloroform, 3,7-dimethyl dodecane, and hexadecane were significantly elevated, but the levels of hexanol and cyclohexanol were distinctly reduced.

Conclusions: This pilot study revealed that the malignant hematological cells could change the components of VOCs in the cell culture flask in a cell type-specific pattern. The traits of VOCs in our setting offered new strategy for hematological malignancies tracing, and would act as potential biomarkers in diagnosis of malignant hematological diseases.

## Background

Acute myeloid leukemia is one of the commonest hematological malignancies with an increasingly occurrence in the past years [1]. Owing to the precision medicine based on the application of prognostic markers and targeted therapy, multidisciplinary approach to patient care, and improved hospital infrastructure, an improved survival has been achieved [2]. However, because of the complex pathogenic mechenism underlying it, the therapy and long-term survival rate in acute myeloid leukemia still needs further improvement [3]. Accurate detection is essential to improve the successful treatment and the long-term survival rate. It is a major issue to be addressed for the diagnosis of acute myelocytic leukemia (AML). Another common hematological malignancy, non-Hodgkin’s lymphoma (NHL), accounts for approximately 4.2% of new diagnosed cancers in the U.S.A., which is the top seventh most commonly diagnosed tumor [4]. NHL consists of heterogeneous entities that vary in biology, clinical behavior, treatment protocol, and disease outcome. The precise diagnosis and intervention reduce cancer-related mortality and improve the quality of life among patients with NHL.

Invasive workup like bone marrow puncture or lymph node biopsy is a basic tool for the diagnosis and outcome evaluation of leukemia and lymphoma. However, these results could be affected by many factors in addition to a time-consuming operating procedure. Furthermore, the traumatic operation and recovery may bring much pain and fear to patients. Therefore, the diagnosis method with the characters of simple, convenient, and cost-effective will be essential for serving the need of accurate and fast diagnosis of leukemia and lymphoma.

Previous studies indicated that more than 2000 compounds were detected in human breath [5], most of them belonged to volatile organic compounds (VOCs) including alkanes, ketones, aldehydes, unsaturated hydrocarbons, alcohols, and aromatic hydrocarbons. Some VOCs were believed to be associated with a pathological state of human body, and the synthesis of VOCs was associated with the environment and genetics. The synthesis of VOCs was involved in the composition of carbon, nitrogen, sulfur, and energy provided by primary metabolism. Thus, the ratio of these blocks affects the concentration of secondary metabolite, such as VOCs, indicating that VOCs have an impact on the metabolite processes. Besides the exhaled gas [6], VOCs were investigated in the headspaces of cancer cell lines [7–9], skin [10], urine [11], and blood [12] normally by gas chromatography–mass spectrometry (GC-MS) technique [13]. Some researches focused on finding the special pattern of VOCs in the exhaled breath or the cell metabolites, which might be used as noninvasive biomarkers to distinguish various diseases such as lung cancer [14,15], colorectal cancer [16], and breast cancer [17,18]. However, up to now, there is no such report in hematological malignant disease.

Solid-phase microextraction (SPME) was widely used in food science, environmental analysis, and medical science [19,20]. The SPME technique was simple, rapid, and renewable without usage of solvent, and it commonly used to collect and preconcentrate the VOCs in the headspace of the culture bottle. Moreover, SPME coupled with GC-MS could improve sensitivity of detection. For example, Sponring et al. [21,22] used an SPME GC-MS analytical technique to identify the specific VOCs for lung cancer cells and normal cells. Their experiment shows that densities of different aldehydes decreased for cancer cells, which is similar to our result. Aldehyde dehydrogenase (ADH) is an important metabolic enzyme *in vivo*. In tumor cells, the enhancement of ADH activity is essential for the growth and metabolism of cells. In squamous cell carcinoma and small cell lung cancer, the activity of ADH 1 family member A1 (ALDH1A1, 1A1) and ADH 3 family member A1 (ALDH3A1, 3A1) was significantly increased. Poli et al. [23] applied SPME-GC-MS as an analytical tool and discovered that the concentration of pentane, toluene, and methylbenzene rose up in the patients with non-small cell lung cancer. They pointed out that the aromatic hydrocarbons may be released by the cancerous tissue. In addition to xylene, other aromatic hydrocarbons released from cancer tissues all presented higher concentration than the normal tissues. In the present study, the SPME sampling technique coupled with GC-MS analysis were used, and our aim was to identify the specific VOCs of JEKO cells and SHI-1 cells.

## Methods

### Cell culture

NHL cell line JEKO was obtained from a pharmacology laboratory of Anhui Medical University. Acute mononuclear leukemia cell line SHI-1 was offered by a hematology laboratory of the first affiliated hospital of Suzhou University. Macrophage cell lines and lymphocyte cell lines, which were the suspended cells in serum-like JEKO and SHI-1, were gifted from a central laboratory of Anhui Medical University affiliated hospital and acted as control. All cells were cultured in RPMI 1640 medium, supplemented with 10% fetal bovine serum, streptomycin (100 mg/l), penicillin (100,000 units/l), and L-glutamine (293 mg/l). The cells were cultivated at 37°C in a humidified atmosphere with 95% air and 5% CO_2_, and the culture medium was refreshed every other day. Three weeks later, those cells in the logarithmic growth phase were used in the following experiment. Macrophages were cultivated as the control group for SHI-1 cells; lymphocytes were serving as the control group for JEKO cells. A medium for the same incubation time and conditions, but without cells, served as a background control. In total, 3.5 × 10^5^ cells per type were plated into the 50 ml glass flask with 5 ml of culture medium. The cells were left in the incubator to cultivate for 24 h and refreshed as scheduled while keeping the culture bottle sealed.

### SPME method and GC-MS analysis

The gas collection was according to the protocol with modification. In brief, the experimental and control tissue-culture flasks were placed on a table with the constant temperature (37°C) for the desired amount of time. Following the sample equilibration, an SPME fiber coated with polydimethylsiloxane (PDMS) was inserted into the headspace of the flasks and kept for 40 min. Then, the SPME syringe was punctured into the sample inlet for the thermal adsorption and desorption (the temperature of adsorption and desorption was 37 and 200°C respectively), where the SPME fiber (the thickness of SPEM fiber was 75 nm) was heated to 180°C and within 2 min by the manufacturer. For the GC-MS operation, the mass spectrometer (TSQ QUANTUM XLS) and chromatographic instrument (TRACE GC ULTRA) were used. Briefly, the column temperature were programmed as follows: started at 50°C for 5 min then ramped at 10°C/min to 230°C, subsequently at 260°C for 5 min according to the manufacture’s instruction of SPME GC-MS (Thermo Fisher Scientific, American). The carrier gas was He (helium) and its flow velocity was 1.0 ml/min. The scan width of MS was 45–250 amu, the temperature of transmission line and ion source was 200°C. The temperature of the quadrupole mass analyzer and the ion source were kept at 150 and 250°C respectively. The split mode was used for injection and purified for 2 min. Before the SPME extraction, the SPME fiber was thoroughly desorbed to remove any possible residual compounds. In our study, all experiments were repeated for 12 times.

### Statistical analysis

In order to eliminate variance from the fluctuation of ionic signals and make the experimental data comparable, we normalized the ionic peak area in every mass spectrometry. Namely, one mass spectra, the peak area of CO_2_ was used as a standard reference and the peak area of certain VOC was counted by *I* ’_m_ = *I*_m_/*I*_CO2_*100 000 000; *I*_m_ represents the raw peak area for the corresponding VOC and *I* ’_m_ is the normalized data. *I*_m_ is the normalized data and represents the raw peak area for the corresponding VOC. Statistical analysis was performed using the Statistical Package for the Social Sciences (SPSS) software version 16 for Windows (SPSS Inc., Chicago, IL, U.S.A.). We applied an one-way analysis of variance (ANOVA) or the Wilcoxon/Kruskal–Wallis one-way analysis of variance to compare the normalized ionic peak area of gas emitted from different groups. A *P*-value of <0.05 was considered as significantly difference. Data were presented as mean ± standard deviation (SD). Graphs were created using GraphPad Prism (version 5.0; GraphPad Software, Inc., La Jolla, CA, U.S.A.) and OriginPro (version 8.0; Microcal Software, Inc., Northampton, MA, U.S.A.).

## Results

### Mass spectrometry comparison of VOCs among the three groups

The typical air chromatograms on VOCs of SHI-1, macrophage cell line, JEKO, lymphocytes cell line, and related blank groups were illustrated in Figures 1 and 2 respectively. A significant difference could be observed in the area of peaks at the same retention time in the cancer, control, and blank groups, which means the different concentrations of the compounds. When compared with the blank group, the peak areas were increased in SHI-1, macrophages, JEKO, and lymphocytes from the exhaled process of cell, and a peak area reduction along with the increase of time might be due to the consumption of nutritional ingredients such as carbon, nitrogen, sulfur as well as energy of medium in cell growth. By means of GC-MS analysis, a total of 20 kinds of VOCs were identified in the SHI-1 system. In total, 8 out of 20 VOCs were found statistically significant, while 2,4-dimethylheptane, benzene, 4-methyl decane, chloroform, 3,7-dimethyl dodecane, and hexadecane detected in the cancer group SHI-1 cell lines exhibit obvious increasing trend, hexanol and cyclohexanol were found dramatically decreased (Table 1). For JEKO cells system, a total of 19 kinds of VOCs were detected, of which nine compounds were found to be significant, while dimethyl sulfide, 2,4-dimethylheptane, methylbenzene, *o*-xylene, dodecane, and 1,3-di-tert-butylbenzene were found to be significantly elevated in the JEKO cell line. Ethanol, hexanal, and benzaldehyde were reduced in their densities (Table 2).

**Figure 1:** Gas chromatograms of VOCs in the headspace of the hematological malignancies cell line SHI-1 (cancer group), macrophage cell line (control group), and blank group.

**Figure 2:** Gas chromatograms of VOCs in the headspace of the hematological malignancies cell line JEKO (cancer group), lymphocyte cell lines (control group), and blank group.

**Table 1:** The comparison of VOCs peak area in the headspace of cancer group (SHI-1cells), control group (human macrophage cells), and medium control (blank group)

Compounds	Mean peak area			*F*/χ^2^	*P* value
	Cancer group	Control group	Blank group		
2,4-Dimethylheptane	1.9449 × 10^7^ ± 5.0014 × 10^6^	5.7271 × 10^6^ ± 4.4027 × 10^6^	0	20.613	0
Benzene	3.2566 × 10^7^ ± 2.3706 × 10^6^	6.3048 × 10^6^ ± 2.3706 × 10^6^	6.2363 × 10^6^ ± 2.2509 × 10^6^	15.680	0
4-Methyl decane	1.6823 × 10^6^ ± 2.7623 × 10^5^	0	0	21.807	0
Chloroform	5.0500 × 10^6^ ± 2.9988 × 10^6^	5.5885 × 10^5^ ± 3.0981 × 10^5^	0	21.256	0
3,7-Dimethyl dodecane	1.2917 × 10^6^ ± 1.6308 × 10^5^	2.7358 × 10^5^ ± 4.5128 × 10^4^	0	21.256	0
Hexanol	0	1.5162 × 10^6^ ± 1.8187 × 10^5^	2.0382 × 10^6^ ± 4.0112 × 10^5^	19.186	0
Cyclohexanol	0	2.9366 × 10^5^ ± 4.3150 × 10^4^	3.8009 × 10^6^ ± 9.1831 × 10^5^	21.256	0
Hexadecane	1.9195 × 10^6^ ± 4.1809 × 10^5^	1.3237 × 10^6^ ± 3.1793 × 10^5^	0	18.931	0

The results were expressed as the mean ± SD. One-way analysis of variance (ANOVA) or the Wilcoxon/Kruskal−Wallis to compare the normalized ionic peak area of gas emitted from three groups.

**Table 2:** The comparison of VOCs peak area in the headspace of cancer group (JEOK cells), control group (human lymphocytes cells), and medium control (blank group)

Compounds	Mean peak area			*F*/χ^2^	*P* value
	Cancer group	Control group	Blank group		
Dimethyl sulfide	9.3692 × 10^7^ ± 1.6314 × 10^7^	0	0	21.807	0
Ethanol	1.0559 × 10^7^ ± 6.3185 × 10^6^	7.1689 × 10^7^ ± 1.9445 × 10^7^	1.1453 × 10^8^ ± 4.5842 × 10^7^	16.485	0
2,4-Dimethylheptane	2.2786 × 10^8^ ± 9.4153 × 10^7^	1.5770 × 10^8^ ± 5.9798 × 10^7^	0	19.017	0
Methylbeneze	2.3378 × 10^8^ ± 9.4232 × 10^7^	1.4177 × 10^8^ ± 5.2523 × 10^7^	9.8781 × 10^7^ ± 7.3435 × 10^7^	6.703	0.006
Hexanal	3.8350 × 10^6^ ± 1.0229 × 10^6^	8.3013 × 10^6^ ± 1.2044 × 10^6^	8.0023 × 10^6^ ± 3.1005 × 10^6^	12.355	0
*o*-Xylene	2.4996 × 10^7^ ± 1.1601 × 10^7^	1.4143 × 10^7^ ± 2.7087 × 10^6^	1.0588 × 10^7^ ± 2.6105 × 10^6^	13.02	0.001
Dodecane	1.0388 × 10^8^ ± 3.1960 × 10^7^	3.9058 × 10^7^ ± 1.2287 × 10^7^	3.3822 × 10^7^ ± 1.0727 × 10^7^	15.605	0
1,3-Di-tert-butylbenzene	2.2445 × 10^8^ ± 3.7074 × 10^7^	1.3091 × 10^8^ ± 5.2283 × 10^7^	1.0075 × 10^8^ ± 5.1086 × 10^7^	15.315	0
Benzaldehyde	2.7386 × 10^7^ ± 1.2392 × 10^7^	5.1230 × 10^7^ ± 1.2347 × 10^7^	7.3170 × 10^7^ ± 1.0903 × 10^7^	29.617	0

The results were expressed as the mean ± SD. One-way analysis of variance (ANOVA) or the Wilcoxon/Kruskal–Wallis to compare the normalized ionic peak area of gas emitted from three groups.

### Comparison of the peak area of VOCs among the three groups

Based on the mass spectral measurements, the distributions of peak areas of the meaningful VOCs from the cancer, control, and blank groups in SHI-1 and JEKO cell lines were displayed in Figures 3 and 4 respectively. From the group of SHI-1 cells, 2,4-dimethylheptane, chloroform, 3,7-dimethyl dodecane, and hexadecane could be detected in the headspace of both SHI-1 and macrophages cell lines, and the peak areas of the former were significantly increased (*P*<0.05). In addition, hexanol and cyclohexanol only appeared in the blank group and control group (*P*<0.05). Benzene occurred in three groups while detectable quantity of benzene increased dramatically in the experimental group (*P*<0.05). To our surprise, 4-methyl decane existed only in the cancer group. After comprehensive analysis of these substances, eight VOCs were found to be significantly different as described above.

**Figure 3:** The peak area distributions of the meaningful eight VOCs for the experimental group SHI-1 cell lines, control group macrophage cell lines, and the blank group. (**A**) 2,4-dimethylheptane, (**B**) benzene, (**C**) 4-methyl decane, (**D**) chloroform, (**E**) 3,7-dimethyl dodecane, (**F**) hexanol, (**G**) cyclohexanol, and (**H**) hexadecane (*n*=8 per group; *P<0.05,**P<0.01).

**Figure 4:** The peak area distributions of the meaningful nine VOCs for experimental group JEKO cell lines, control group lymphocyte cell lines, and the blank group. (**A**) dimethyl sulfide, (**B**) ethanol, **(C**) 2,4-dimethylheptane, (**D**) methylbenzene, (**E**) hexanal, (**F**) *o*-xylene, (**G**) dodecane, (**H**) 1,3-di-tert-butylbenzene, and (**I**) benzaldehyde; (*n*=8 each group; **P<0.01, *P<0.05).

In the group of JEKO cell line, the particular common identified VOCs in the headspace of tissue culture bottle of three groups were ethanol, methylbeneze, hexanal, *o*-xylene, dodecane,1,3-di-tert-butylbenzene, and benzaldehyde. Dimethyl sulfide and 2,4-dimethylheptane were not been detected in the blank group. Surprisingly, dimethyl sulfide only existed in the experimental group. From the chart, we found that the densities of ethanol, hexanal, and benzaldehyde in JEKO cells were significantly decreased, while the concentration of other compounds was relatively higher.

## Discussion

SPME is an exhaustive sample preparation technique that was much perfect than other traditional sample preparation techniques, such as low organic solvent consumption. In the last few years, the introduction of SPME has acquired great progress in the sample preparation area [24]. Recently, extraction procedures using SPME, followed by GC–MS, have been widely used in VOCs research [25]. From this study, the SPME method was employed for the analysis of VOCs, which was essential for the detection of cancer markers in clinical practice.

According to the definition of the World Health Organization (WHO), VOCs refer to some organics with the boiling points between 50 and 250°C, and their components consist of the carbon number between C6 and C16. Normally, the VOCs mainly included alkanes, alkenes, ketones, aromatic hydrocarbons, terpenes, and siloxanes [26]. The breath sample testing has been attempted to diagnose diseases for approximately 30 years [27]. In recent years, many studies tried to propose them for the tumor diagnosis, and found that the VOCs exhaled by different patients were diverse, especially in lung cancer research [28,29]. To our knowledge, neither human breath nor cell lines related with VOCs analysis in hematological malignancy has been reported in literature.

Human exhaled VOCs include exogenous and endogenous components. The exogenous VOCs refer to environmental air that enter the body by breathing or through skin absorption, and finally passes through alveoli to be excreted. As for the endogenous VOCs, previous study suggested that they were produced through the process of oxidative stress in the body [30,31], which were relatively stable and had low solubility in blood. Endogenous VOCs were associated with the body lesions, which were the compounds that could be detected in human breath. As a result of low concentration of those VOCs, some special pretreatment techniques and high sensitivity instruments such as SPME GC–MS, proton transfer reaction-mass spectrometry (PTR-MS), and electronic nose sensors are needed for accurate detection. For the abnormality of hematopoiesis or the blood cells distribution, any organs and tissues throughout the body almost can be infringed. The high metabolism status of tumor cells can lead to changes of the endogenous VOCs. Breath analysis has qualitative and quantitative analysis potential to trace VOCs by diseases. In addition, breath samples are obtainable, non-invasive, and cost-effective in regards to analysis. All these made exhaled gas considerably attractive in tumor diagnosis. In the present study, the experimental group of SHI-1 and JEKO cells was found with a characteristic VOCs phenotype. In our study, the aromatic VOCs and alkanes were also significantly increased. This suggests that the activity of oxygen free radical in blood cancer cells is enhanced, which might cause lipid peroxidation and lead to cell membrane damage. The unsaturated fatty acid degradation is also increased; thus, the VOCs are increased when compared with the normal cells. Moreover, Ucar et al. [32] reported that the activity of ADH could be used as a marker for lung cancer. As we all know, ethanol is degraded by alcohol dehydrogenase to produce acetaldehyde, and methanol is degraded to formaldehyde. Aldehydes that are formed in the body are oxidized by ADH to yield carboxylic acids. It is speculated that the reduction of these alcohols and aldehydes in headspace gas of culture bottle cultivated SHI-1 cells, and JEKO cells may be related to the increased activity of ADH in the tumor cells. But the ultimate mechanism still needs to be further elucidated.

Previous researches have shown that the alteration of genes expression for cytochrome 450 mixed enzyme system in cancer patients, which might cause the metabolites degraded by increasing oxidative stress, including alkane and single methyl alkane, leading to changes in components of VOCs [33–35]. It was part of the mechanism of the VOCs production in hematological malignancy. Wang et al. [36] has analyzed VOCs in exhaled breath, lung cancer tissues, and cell lines. Comparing with the results, 2-pentade canone and nonadecane were the mutual VOCs for three groups, but the composition of VOCs in exhaled breath is more complex than in lung cancer cells and tissues. This indicated that the metabolism of VOCs* in vivo* was more complicated than *in vitro*. The metabolism of the body-like methylation may make a contribution for the structure change of the VOCs, but there still existed some relationship between them. The VOCs are not produced by the single factor. At present, we have analyzed VOCs from cell line of hematological malignancies and found that the VOCs had statistically significant difference compared with the control group, showing that the VOCs may be potential markers for hematological malignancy. The mechanism *in vivo* perspective remains to be further studied.

## Conclusions

To analyze an exhaled gas sample, one can find many different techniques and methods [36,37]. This study has detected VOCs in metabolic products of leukemia cells and lymphoma cells, and has screened out statistically significant difference of VOCs, suggesting these specific VOC substances may be potential markers of leukemia cells and lymphoma cells. Multiple-sample research was performed to verify the existing data and to explore the mechanism of endogenous VOCs production of different types of cancer. The detection of volatile markers from exhaled gas analysis shed new light for the diagnosis of patients with leukemia and lymphoma.

## Abbreviations

ADH: aldehyde dehydrogenase
NHL: non-Hodgkin’s lymphoma
SPME: solid-phase microextraction
VOC: volatile organic compound
GC-MS: gas chromatography-mass spectrometry

## References

[1] ZeunerA., PediniF., SignoreM., RuscioG., MessinaC., TafuriA. (2006) Increased death receptor resistance and FLIPshort expression in polycythemia vera erythroid precursor cells. Blood 107, 3495–35021638493010.1182/blood-2005-07-3037

[2] RobozG.J. (2011) Novel approaches to the treatment of acute myeloid leukemia. Hematol. Am. Soc. Hematol. Educ. Program 2011, 43–5010.1182/asheducation-2011.1.4322160011

[3] DerolfA.R., KristinssonS.Y., AnderssonT.M., LandgrenO., DickmanP.W. and BjorkholmM. (2009) Improved patient survival for acute myeloid leukemia: a population-based study of 9729 patients diagnosed in Sweden between 1973 and 2005. Blood 113, 3666–36721902030610.1182/blood-2008-09-179341

[4] ChiuB.C. and HouN. (2015) Epidemiology and etiology of non-hodgkin lymphoma. Cancer Treat. Res. 165, 1–252565560410.1007/978-3-319-13150-4_1

[5] PhillipsM. (1992) Breath tests in medicine. Sci. Am. 267, 74–79150251110.1038/scientificamerican0792-74

[6] XuZ.Q., BrozaY.Y., IonsecuR., TischU., DingL., LiuH. (2013) A nanomaterial-based breath test for distinguishing gastric cancer from benign gastric conditions. Br. J. Cancer 108, 941–9502346280810.1038/bjc.2013.44PMC3590679

[7] BarashO., PeledN., TischU., BunnP.A., HirschF.R. and HaichH. (2012) Classification of lung cancer histology by gold nanoparticle sensors. Nanomedicine 8, 580–5892203308110.1016/j.nano.2011.10.001PMC4745892

[8] MochalskiP., SponringA., KingJ., UnterkoflerK., TroppmairJ. and AmannA. (2013) Release and uptake of volatile organic compounds by human hepatocellular carcinoma cells (HepG2) in vitro. Cancer Cell Int. 13, 722387048410.1186/1475-2867-13-72PMC3717104

[9] FilipiakW., SponringA., FilipiakA., AgerC., SchubertJ., MiekischW. (2010) TD-GC-MS analysis of volatile metabolites of human lung cancer and normal cells in vitro. Cancer Epidemiol. Biomarkers Prev. 19, 182–1952005663710.1158/1055-9965.EPI-09-0162

[10] D'AmicoA., BonoR., PennazzaG., SantonicoM., MantiniG., BernabeiM. (2008) Identification of melanoma with a gas sensor array. Skin Res. Technol. 14, 226–2361841256710.1111/j.1600-0846.2007.00284.x

[11] HanaiY., ShimonoK., MatsumuraK., VachaniA., AlbeldaS., YamazakiK. (2012) Urinary volatile compounds as biomarkers for lung cancer. Biosci. Biotechnol. Biochem. 76, 679–6842248493010.1271/bbb.110760

[12] XueR., DongL., ZhangS., DengC., LiuT., WangJ. (2008) Investigation of volatile biomarkers in liver cancer blood using solid-phase microextraction and gas chromatography/mass spectrometry. Rapid Commun. Mass Spectrom. 22, 1181–11861835056210.1002/rcm.3466

[13] MoserB., BodrogiF., EiblG., LechnerM., RiederJ. and LirkP. (2005) Mass spectrometric profile of exhaled breath–field study by PTR-MS. Respir. Physiol. Neurobiol. 145, 295–3001570554310.1016/j.resp.2004.02.002

[14] PhillipsM., CataneoR.N., CumminA.R., GagliardiA.J., GleesonK., GreenbergJ. (2003) Detection of lung cancer with volatile markers in the breath. Chest 123, 2115–21231279619710.1378/chest.123.6.2115

[15] FilipiakW., FilipiakA., SponringA., SchmidT., ZelgerB., AgerC. (2014) Comparative analyses of volatile organic compounds (VOCs) from patients, tumors and transformed cell lines for the validation of lung cancer-derived breath markers. J. Breath Res. 8, 0271112486210210.1088/1752-7155/8/2/027111

[16] WangC., LiP., LianA., SunB., WangX., GuoL. (2014) Blood volatile compounds as biomarkers for colorectal cancer. Cancer Biol. Ther. 15, 200–2062410061210.4161/cbt.26723PMC3928136

[17] MetcalfeE and EtizD. (2016) Early transient radiation-induced brachial plexopathy in locally advanced head and neck cancer. Contemp. Oncol. (Pozn.) 20, 67–722709594310.5114/wo.2015.55876PMC4829741

[18] DiasJ.A., FredriksonG.N., EricsonU., GullbergB., HedbladB., EngstromG. (2016) Low-grade inflammation, oxidative stress and risk of invasive post-menopausal breast cancer - a nested case-control study from the malmo diet and cancer cohort. PLoS ONE 11, e01589592739132410.1371/journal.pone.0158959PMC4938491

[19] SajidM., BasheerC., NarasimhanK., ChoolaniM. and LeeH.K. (2015) Application of microwave-assisted micro-solid-phase extraction for determination of parabens in human ovarian cancer tissues. J. Chromatogr. B Analyt. Technol. Biomed. Life Sci. 1000, 192–19810.1016/j.jchromb.2015.07.02026245364

[20] ZhaoQ., LuQ. and FengY.Q. (2013) Dispersive microextraction based on magnetic polypyrrole nanowires for the fast determination of pesticide residues in beverage and environmental water samples. Anal. Bioanal. Chem. 405, 4765–47762351560810.1007/s00216-013-6866-5

[21] SponringA., FilipiakW., MikovinyT., AgerC., SchubertJ., MiekischW. (2009) Release of volatile organic compounds from the lung cancer cell line NCI-H2087 in vitro. Anticancer Res. 29, 419–42619331181

[22] SponringA., FilipiakW., AgerC., SchubertJ., MiekischW., AmannA. (2010) Analysis of volatile organic compounds (VOCs) in the headspace of NCI-H1666 lung cancer cells. Cancer Biomark 7, 153–1612126319110.3233/CBM-2010-0182PMC12922879

[23] PoliD., CarbognaniP., CorradiM., GoldoniM., AcampaO., BalbiB. (2005) Exhaled volatile organic compounds in patients with non-small cell lung cancer: cross sectional and nested short-term follow-up study. Respir. Res. 6, 711601880710.1186/1465-9921-6-71PMC1185565

[24] BoyaciE., Rodriguez-LafuenteA., GorynskiK., MirnaghiF., Souza-SilvaE.A., HeinD. (2015) Sample preparation with solid phase microextraction and exhaustive extraction approaches: Comparison for challenging cases. Anal. Chim. Acta 873, 14–302591142610.1016/j.aca.2014.12.051

[25] HeM., YangZ.F., GuanW.N., Vicente GoncalvesC.M., NieJ. and WuH. (2016) GC-MS analysis and volatile profile comparison for the characteristic smell from liang-wai gan cao (glycyrrhiza uralensis) and honey-roasting products. J. Chromatogr. Sci. 54, 879–8872699411310.1093/chromsci/bmw034

[26] SchleibingerH., LaussmannD., BrattigC., ManglerM., EisD. and RudenH. (2005) Emission patterns and emission rates of MVOC and the possibility for predicting hidden mold damage? Indoor Air 15, 98–1041591053510.1111/j.1600-0668.2005.00349.x

[27] BuszewskiB., UlanowskaA., KowalkowskiT. and CieslinskiK. (2011) Investigation of lung cancer biomarkers by hyphenated separation techniques and chemometrics. Clin. Chem. Lab. Med. 50, 573–5812203513910.1515/CCLM.2011.769

[28] PengG., HakimM., BrozaY.Y., BillanS., Abdah-BortnyakR., KutenA. (2010) Detection of lung, breast, colorectal, and prostate cancers from exhaled breath using a single array of nanosensors. Br. J. Cancer 103, 542–5512064801510.1038/sj.bjc.6605810PMC2939793

[29] Wong RP., FlemattiG.R. and DavisT.M. (2012) Investigation of volatile organic biomarkers derived from Plasmodium falciparum in vitro. Malar. J. 11, 3142295846010.1186/1475-2875-11-314PMC3468367

[30] KimJ.H., MoonJ.Y., ParkE.Y., LeeK.H. and HongY.C. (2011) Changes in oxidative stress biomarker and gene expression levels in workers exposed to volatile organic compounds. Ind. Health 49, 8–142082363910.2486/indhealth.ms1112

[31] Caliskan-CanE., FiratH., ArdicS., SimsekB., TorunM. and Yardim-AkaydinS. (2008) Increased levels of 8-hydroxydeoxyguanosine and its relationship with lipid peroxidation and antioxidant vitamins in lung cancer. Clin. Chem. Lab. Med. 46, 107–1121819408210.1515/CCLM.2008.010

[32] UcarD., CogleC.R., ZucaliJ.R., OstmarkB., ScottE.W., ZoriR. (2009) Aldehyde dehydrogenase activity as a functional marker for lung cancer. Chem. Biol. Interact. 178, 48–551895207410.1016/j.cbi.2008.09.029PMC2976869

[33] ShahP.P., SinghA.P., SinghM., MathurN., MishraB.N., PantM.C. (2008) Association of functionally important polymorphisms in cytochrome P4501B1 with lung cancer. Mutat. Res. 643, 4–101857350810.1016/j.mrfmmm.2008.05.001

[34] HassaneinM., CallisonJ.C., Callaway-LaneC., AldrichM.C. and GroganE. (2012) The state of molecular biomarkers for the early detection of lung cancer. Cancer Prev. Res. (Phila) 5, 992–10062268991410.1158/1940-6207.CAPR-11-0441PMC3723112

[35] WangC., KeC., WangX., ChiC., GuoL., LuoS. (2014) Noninvasive detection of colorectal cancer by analysis of exhaled breath. Anal. Bioanal. Chem. 406, 4757–47632482006210.1007/s00216-014-7865-x

[36] WangY., HuY., WangD., YuK., WangL., ZouY. (2012) The analysis of volatile organic compounds biomarkers for lung cancer in exhaled breath, tissues and cell lines. Cancer Biomark 11, 129–1372314415010.3233/CBM-2012-00270PMC13016210

[37] CheH., WortmannA., ZhangW. and ZenobiR. (2007) Rapid in vivo fingerprinting of nonvolatile compounds in breath by extractive electrospray ionization quadrupole time-of-flight mass spectrometry. Angew. Chem. Int. Ed. Engl. 46, 580–5831708047110.1002/anie.200602942

